# Modified box dimension and average weighted receiving time on the weighted fractal networks

This article has been retracted.

**DOI:** 10.1038/srep18210

**Published:** 2015-12-15

**Authors:** Meifeng Dai, Yanqiu Sun, Shuxiang Shao, Lifeng Xi, Weiyi Su

**Affiliations:** 1 Nonlinear Scientific Research Center, Faculty of Science, Jiangsu University Zhenjiang, Jiangsu, 212013, P.R. China; 2 Institute of Mathematics, Zhejiang Wanli University, Ningbo 315100, P.R. China; 3 Department of Mathematics, Nanjing University, Nanjing, 210093, P. R. China

## Abstract

In this paper a family of weighted fractal networks, in which the weights of edges have been assigned to different values with certain scale, are studied. For the case of the weighted fractal networks the definition of modified box dimension is introduced, and a rigorous proof for its existence is given. Then, the modified box dimension depending on the weighted factor and the number of copies is deduced. Assuming that the walker, at each step, starting from its current node, moves uniformly to any of its nearest neighbors. The weighted time for two adjacency nodes is the weight connecting the two nodes. Then the average weighted receiving time (AWRT) is a corresponding definition. The obtained remarkable result displays that in the large network, when the weight factor is larger than the number of copies, the AWRT grows as a power law function of the network order with the exponent, being the reciprocal of modified box dimension. This result shows that the efficiency of the trapping process depends on the modified box dimension: the larger the value of modified box dimension, the more efficient the trapping process is.

Recently, self-similar fractals have attracted much attention. The renormalization procedure tiles a network according to the box-covering algorithm. Self-similarity is then obtained if the network structure remains invariant under the renormalization. Gallos *et al.* reviewed the findings of self-similarity in complex networks. Using the box-covering technique, it was shown that many networks present a fractal behavior, which is seemingly in contrast to their small-world property^1^. Then they used scaling theory to quantify the degree of correlations in the particular case of networks with a power-law degree distribution^2^. Starting from the fractal network, Rozenfeld *et al.*^3^ applied renormalization group theory to study complex networks using the box covering technique, which is useful to classify network topologies into universality classes in the space of configurations. After defining a unified mathematical framework for both immunization and spreading, Morone and Makse provided its optimal solution in random networks by mapping the problem onto optimal percolation and found that the top influencers are highly counterintuitive^4^.

Motivated by the hierarchial and scale-free networks^5^,^6^, Komj*á*thy and Simon^7^ introduced deterministic the scale-free graphs derived from a graph directed self-similar fractal. Chen *et al.*^8^ constructed a class of scale-free networks with fractal structure based on the subshift of finite type and base graphs. When embedding the growing network into the plane, its image is a graph-directed self-affine fractal, whose Hausdorff dimension is related to the power law exponent of cumulative degree distribution.

Unfortunately, many previous works have focused on the un-weighted networks. In real networks, the relations between two nodes have been affected by specific physical properties of network elements, including the number of passengers traveling yearly between two airports in airport networks^9^, to the intensity of predator-prey interactions in ecosystems^10^ or the traffic measured in packets per unit time between routers in the Internet^11^. So weighted networks commendably represent the natural framework to describe natural, social, and technological systems, in which the intensity of a relation or the traffic between elements is an important parameter^12^,^13^. In general terms, weighted networks are extension of networks or graphs^14^,^15^, in which each edge between nodes *i* and *j* is associated with a variable , called the weight.

A key quantity related to weighted networks is the mean weighted first-passage time (MWFPT), that is, the expected weighted first time for the walker starting from a source node to a given target node. The average weighted receiving time (AWRT) is the sum of mean weighted first-passage times (MFPTs) for all nodes absorpt at the trap located at a given target node^16^,^17^,^18^. In 2013, Dai *et al.* introduced the non-homogenous weighted Koch networks depending on the three weight factors^19^. They defined the average weighted receiving time (AWRT) for the first time and studied the AWRT on random walk. Recently, fractals have also attracted an increasing attention in physics and other scientific fields, owning to the striking beauty intrinsic in their structures and the significant impact of the idea of fractals. These structures have been a focus of research objects and many underlying properties have been found. So it makes sense to combining weighted networks with fractals which are called weighted fractal networks. Daudert and Lapidus^20^ studied weighted graphs and random walks on the Koch snowflake. Carletti and Righi^21^ defined a class of weighted complex networks whose topology can be completely analytically characterized in terms of the involved parameters and of the fractal dimension.

This paper is organized as follow. Based on weighted fractal networks^21^, we introduce a family of the weighted fractal networks depending on the number of copies *s* and the weight factor *r* in the next section. In Section 3, the definition of modified box dimension and a rigorous proof for its existence are given in the case of the weighted fractal networks. In Section 4, the average weighted receiving time (AWRT) on random walk is obtained by recursive formulas for  and . When the weight factor is larger than the number of copies, we show that the efficiency of the trapping process depends on the modified box dimension: the larger the value of modified box dimension, the more efficient the trapping process is. In the last section we draw conclusions.

## Weighted fractal networks

In this section a family of weighted fractal networks are introduced.

Let  be a positive real numbers, and  be a positive integer.

(1) Let  be our base graph, composed by  nodes . We partition  into two non-empty sets , labeled attaching node,  all other nodes except for the attaching node, satisfying the symmetry of nodes in . The edge set of  is denoted by . If the pair  is connected by an edge, then this edge is denoted by . Each of  with unit weight.

**Remark:** The symmetry of nodes  in  means that the network  is invariable no matter how two arbitrary nodes *i* and *j* are exchanged .

(2) For any ,  is obtained from  (see Fig. 1):  has one attaching node labelled by . Let  be *s* copies of .  is obtained by the union of *s* copies . Let  be the set of nodes in , which is . If the pair  is connected by an edge, then this edge is denoted by . Let  be the set of edges in . For  let us denote by  the node in  image of the labeled node . Let , then link all those label nodes to the attaching node , each of the edges  assigns weight .

The weighted fractal networks are set up.

According to the construction of the weighted fractal networks, one can see that , the weighted fractal networks of *n*- th generation, is characterized by three parameters *n*, *s* and *r*: *n* being the number of generations, *s* being the number of copies, and *r* representing the weight factor. The total number of nodes in  is as follows.



## Modified box dimension

**Definition 3.1.** The weighted shortest path of nodes *i* and *j* in the weighted graphs  is given by



where Γ is the set of paths linking *i* and *j* in 21.

The self-similar property of real-world networks, box-counting method turns to be practical^22^. The method works as follows: we partition the nodes into boxes of size . The maximal distance between vertices within a box is at most . The resulting number of boxes needed to tile the networks denoted by . Then the box dimension  is defined by .

Modified box dimension was motivated by the fact that in the case of the weighted fractal networks the original definition of box dimension is infinite. It is worth mentioning, our new concept of dimension does exist and is finite for this model as Theorem 3.3 shows.

**Definition 3.2.** The modified box dimension is defined by



where  and  denotes the minimal number of boxes of size  that we need to cover .

**Theorem 3.3.** For the weighted fractal networks the modified box dimension:



where *s* is the number of copies, *r* is the weighted factor.

For convenience of description, we recall the following notations.

(i) Let  be the set of nodes in , which is  where , and  be the set of edges in .

(ii) Given , we denote the common prefix by  s.t.  and .

(iii) We fix an arbitrary self-map *p* of  such that for , , i.e., .

For a word , we define



Then  is an edge in .

## The diameter of *G*_*n*_

**Lemma 3.4.** The diameter of  is



**Proof.** We will prove this from two respects.

(1) Considering the worst case scenario, i.e., choosing  and  such that (i) . (ii) , yields that



(2) We construct a path  between two arbitrary nodes *x* and *y* that is no longer than . Let  where  and , where .

Starting from *x* the first half of the path  is as follows:



Starting from ***y*** the first half of the path  is as follows.



In this way



Clearly,



## Lower bound of modified box dimension

**Lemma 3.5.** The following inequality holds for ,



**Proof.** It is easy to see that we need one *l*_1_-box to cover . It follows from the weighted structure of  that  contains  copies of  and  nodes. This implies that we can cover  with  *l*_1_-boxes. #

**Lemma 3.6.**



**proof.** Suppose that  and  two arbitrary nodes in  contained by the same *l*_1_-box, i.e., the distance between *x* and *y* is not greater than . If we blow them up, we get two cylinder sets of nodes:



and



Next, we calculate the maximal distance between the elements of ***X*** and ***Y***. Considering the worst case scenario ,  and . Namely that



and



Starting from  it at most takes  steps to reach the . Similarly, starting from  we need at most  steps to reach .

Thus the distance between  and  is not greater than . Therefor, the same -boxing that we have used in  is an appropriate -boxing for . #

From Eqs (4) and (5), we can see that  Then from Eqs (1, 2, 3), we obtain



## Upper bound of modified box dimension

**Lemma 3.7.** The following inequality holds for 



**Proof.** For every digit , we define the cylinder set  of words  with .

Let . Now we give a lower bound on the shortest path between  and  thus we need at least  steps on any path between  and . These witness must be in distinct  boxes, so we need at least  *l*_1_-boxes to cover . *#*

**Lemma 3.8.** The following inequality holds



**Proof.** We have constructed  nodes in  whose pairwise distance is greater than . It is enough to show that we can find the same number of nodes (i.e., ) in ,  such that the pairwise distances between them are greater than , this implies



Let



where the cylinder set of nodes



Now we give a lower bound on the shortest path between  and  where . We need at least  steps on any path between  and . Hence these witness must be in distinct  boxes. So we need at least  -boxes to cover . i.e., substitutily  and  yields that



From Eq. (7) we can see that . Then from Eqs (1, 2, 3), we obtain



**Proof of Theorem 3.3.** Combining lower bound and upper bound of modified box dimension i.e., Eqs (6) and (8) yields Theorem 3.3, hence:



## The average weighted receiving time on random walk

The purpose of this section is to determine explicitly the average weighted receiving time (AWRT)  and to show how  scales with network order. We aim at a particular case on  with the trap placed on the attaching node , let us denote by 0. All other nodes, except for the attaching node, are denoted by .

Assuming that the walker, at each step, starting from its current node, moves uniformly to any of its nearest neighbors.

For two adjacency nodes *i* and *j*, the weighted time is defined as the corresponding edge weight . The mean weighted first-passing time (MWFPT) is the expected first arriving weighted time for the walks starting from a source node to a given target node. Let  be the mean weighted first-passage time (MWFPT) for a walker starting from Node *i* to Node *j*. Let  be the MWFPT from Node *i* to the trap.  is the average weighted receiving time (AWRT), which is defined as the average of  over all starting nodes other than the trap.  is the key question concerned in this paper.

**Theorem 4.1.** For a large system, i.e., ,

(1) if , we have the following expression for the dominating term of :



where ;

(2) if , we have the following expression for the dominating term of :



(3) if , we have the following expression for the dominating term of :



**Remark.** This confirms that in the large  limit, if  then the AWRT grows as a power law function of the network order with the exponent, represented by , being the reciprocal of . When  grows from 0 to 1, the exponent decreases from  approaches 1. This also means that the efficiency of the trapping process depends on the modified box dimension: the larger the value of modified box dimension, the more efficient the trapping process is.

**Proof.** By definition,  is given by



Here, we denote by  the sum of MWFPTs for all nodes to absorption at the trap located the attaching node , i.e.,



Thus, the problem of determining  is reduced to finding . We will compute  by segmenting .

From the self-similarity construction method of ,  can be regarded as merging  groups, sequentially denoted by . The  groups are obtained as follows.  includes the central Node 0 and *s* nodes denoted by ,  Each node in *s* nodes is linked to the central Node 0 through the weighted time ;  is a copy of . In order to completely explain the division of the general weighted fractal networks, we present the special division of the ‘Sierpinski’ weighted fractal networks when  (see Fig. 2).

Through this division, we can rewrite the sum  as follows:





where .

Thus, the problem of determining  is reduced to finding . Note that the strength of Node  is  according to the construction of . Using the division of , we have



Through the reduction of Eq. (13), we obtain



In the given initial network , let  be the the mean weighted first-passage times (MWFPTs) for a walker from Node *i* in  to the attaching node 0 in . Here, we denote by  the sum of MWFPTs for all nodes to the attaching node 0, i.e., . Because of the symmetry of nodes ,  and .  is a constant number for the given initial network . Considering the initial network , one can prove



Through the simplifications of Eq. (15), we obtain



From Eq. (16), we can solve Eq. (14) recursively to yield



Using the construction of , we have



When  from Eqs (17) and (18), we can solve Eq. (10) inductively to yield



Hence, , which we are concerned about, could be expressed as follows:



(1) If , the dominating term of  is written as follows:



For a large system, i.e., , from Eq. (1) we have the following expression for the dominating term of 



where .

(2) If , the dominating term of  is written as follows:



For a large system, i.e., , from Eq. (1) we have the following expression for the dominating term of :



(3) If *r* = *s*, from Eqs (17) and (18), we can solve Eq. (12) inductively to yield



For a large system, i.e., , from Eq. (1) we have the following expression for the dominating term of :



## Conclusions

In this paper, we introduced a family of weighted fractal networks with weight factor *r*. We mainly studied its modified box dimension and AWRT on the weighted fractal networks. For the case of , the AWRT grows as a power law function of the network order with the exponent, being the reciprocal of . We found that when  grows from 0 to 1, the exponent decreases from  approaches 1. This result showed that the efficiency of the trapping process depends on the modified box dimension: the larger the value of modified box dimension, the more efficient the trapping process is. Otherwise, for the case of , the AWRT grows linearly with the network size , and for the case of , the AWRT grows with increasing order  as .

It should be mentioned that we only studied a particular family of weighted fractal networks, whether the conclusion also holds for other more general networks, which needs further investigation.

## Additional Information

**How to cite this article**: Dai, M. *et al.* Modified box dimension and average weighted receiving time on the weighted fractal networks. *Sci. Rep.* **5**, 18210; doi: 10.1038/srep18210 (2015).

## Figures and Tables

**Figure 1:** Take the ‘Cantor dust’ weighted fractal networks for example.

**Figure 2:** Take the ‘Sierpinski’ weighted fractal networks *G*_*n*_, for example, *G*_2_ is regarded as merging , , , .
